# Muscle fatigue: general understanding and treatment

**DOI:** 10.1038/emm.2017.194

**Published:** 2017-10-06

**Authors:** Jing-jing Wan, Zhen Qin, Peng-yuan Wang, Yang Sun, Xia Liu

**Affiliations:** 1 Department of Pharmacology, School of Pharmacy, Second Military Medical University, Shanghai, China

## Abstract

Muscle fatigue is a common complaint in clinical practice. In humans, muscle fatigue can be defined as exercise-induced decrease in the ability to produce force. Here, to provide a general understanding and describe potential therapies for muscle fatigue, we summarize studies on muscle fatigue, including topics such as the sequence of events observed during force production, *in vivo* fatigue-site evaluation techniques, diagnostic markers and non-specific but effective treatments.

## Introduction

Fatigue is a common non-specific symptom experienced by many people and is associated with many health conditions. Often defined as an overwhelming sense of tiredness, lack of energy and feeling of exhaustion, fatigue relates to a difficulty in performing voluntary tasks.^1^ Fatigue accumulation, if not resolved, leads to overwork, chronic fatigue syndrome (CFS), overtraining syndrome, and even endocrine disorders, immunity dysfunction, organic diseases and a threat to human health.

There are many different fatigue classification methods. According to its duration, fatigue can be classified into acute fatigue and chronic fatigue. Acute fatigue can be quickly relieved by rest or life-style changes, whereas chronic fatigue is a condition defined as a persistent tiredness lasting >months that is not ameliorated by rest.^2, 3, 4^ Fatigue can also be classified as mental fatigue, which refers to the cognitive or perceptual aspects of fatigue, and physical fatigue, which refers to the performance of the motor system.^1^

Muscle fatigue is defined as a decrease in maximal force or power production in response to contractile activity.^5^ It can originate at different levels of the motor pathway and is usually divided into central and peripheral components. Peripheral fatigue is produced by changes at or distal to the neuromuscular junction. Central fatigue originates at the central nervous system (CNS), which decreases the neural drive to the muscle.^5, 6^ Muscle fatigue is a commonly experienced phenomenon that limits athletic performance and other strenuous or prolonged activity. It is also increases and restricts daily life under various pathological conditions, including neurological, muscular and cardiovascular disorders, as well as aging and frailty. This review primarily focuses on muscle fatigue, particularly during intense exercise, to provide a basic understanding and potential therapies for muscle fatigue.

## Factors that affect muscle contraction and fatigue

The production of skeletal muscle force depends on contractile mechanisms, and failure at any of the sites upstream of the cross-bridges can contribute to the development of muscle fatigue, including nervous, ion, vascular and energy systems.^7^ Specifically, metabolic factors and fatigue reactants during the process of contraction, such as hydrogen (H^+^) ions, lactate, inorganic phosphate (Pi), reactive oxygen species (ROS), heat shock protein (HSP) and orosomucoid (ORM), also affect muscle fatigue.

### Neural contributions

Central neurotransmitters, especially 5-HT, DA and NA, play important role during whole-body exercise and fatigue. 5-HT produces a negative effect, whereas methylphenidate, a DA-releasing enhancer and reuptake inhibitor, produces a positive effect in exercise performance.^8^ The so-called central fatigue hypothesis states that exercise induces changes in the concentrations of these neurotransmitters, and fatigue arises from changes within the CNS (or proximal to the neuromuscular junction). However, recent data have shown that drugs influencing the neurotransmitter systems scarcely perturb performance under normal ambient temperatures but significantly improve endurance under high ambient temperatures. For example, the NA reuptake inhibitor reboxetine and a dual DA/NA reuptake inhibitor, bupropion, have a negative effect^9, 10, 11^ on exercise performance under normal temperature. However, under heat, reboxetine decreases, whereas bupropion increases performance, thus suggesting that the thermoregulatory system may have an important influence on exercise performance.

The CNS, via a central neurotransmitter, produces various excitatory and inhibitory inputs on the spinal motoneurons, thus ultimately activating motor units (MUs) to achieve the force output. The strength and timing of contraction are controlled by the firing of the motoneurons. When first recruited in a healthy system, MUs usually fire at 5–8 Hz. During brief nonfatiguing voluntary contractions in humans, the mean MU firing rates are 50–60 Hz.^12^ MUs are recruited or derecruited in an orderly fashion on the basis of the motoneuron size, and they essentially control the amount of muscle tissue being activated.^13^

Slowing or cessation of MU firing contributes to the loss of force that marks fatigue. Motoneuron firing is influenced by intrinsic changes in the motoneuron properties, descending drive and afferent feedback. During fatiguing maximal contractions, motoneuron firing rates decrease because of the following factors: (1) Repetitive activation (repeated firing) of motoneurons leads to a decrease in their excitability to excitatory synaptic input;^14^ (2) the excitatory drive from the motor cortex or other supraspinal area to the motoneurons is lower;^14^ (3) the firing of group III/IV muscle afferents is increased,^15, 16^ thus decreasing motoneuron firing; (4) the firing of muscle spindles (sensory receptors) is decreased, thus decreasing firing of group Ia muscle afferents, increasing presynaptic inhibition, and finally decreasing motoneuron firing;^17, 18^ (5) specifically, group III/IV muscle afferents also exhibit feedback interaction with cardiovascular and respiratory processes via the autonomic nervous system, thereby improving muscle blood flow and oxygenation and consequently slowing the development of fatigue of the muscle itself.^14^

### Ca^2+^

Neural activation results in signal transmission from the brain to the muscle’s transverse tubules, inducing calcium release from the sarcoplasmic reticulum (SR) into the cytosol and initiation of cross-bridge cycling. This excitation-contraction coupling process involves the following events: the action potential (AP) is generated at the neuromuscular junction and propagates along the surface membrane and into the transverse tubules, where it is detected by voltage-sensor molecules (the dihydropyridine receptors, VS/DHPRs), which in turn open the ryanodine receptor-Ca^2+^ release channels (RyR1 isoform in skeletal muscle) in the adjacent SR and cause release of Ca^2+^ into the sarcoplasm.^19^ The binding of Ca^2+^ to troponin moves tropomyosin away from the myosin-binding site on actin, thus permitting cross-bridge cycling. The removal of Ca^2+^ from the cytoplasm by Ca^2+^ ATPase results in the recovery of tropomyosin to its blocked position, and relaxation occurs.^20^

Impaired calcium release from the SR has been identified as a contributor to fatigue in isolated skeletal muscle fibers. Several possible mechanisms have been proposed: (1) AP involves Na^+^ influx, and the subsequent repolarization involves K^+^ efflux in muscle cells. High-frequency stimulation may lead to extracellular K^+^ accumulation, which may decrease voltage sensor activation and the action potential amplitude; (2) Most of the ATP in a rested fiber is Mg^2+^ bound. Fatigue can induce a decrease in intracellular ATP and an increase in free Mg^2+^, thus decreasing the effectiveness of SR Ca^2+^ channel opening; (3) Exposure to myoplasmic phosphate causes a sustained decrease in SR Ca^2+^ release in skinned fiber because inorganic phosphate can enter the SR and precipitate Ca^2+^, thus decreasing the free Ca^2+^ and amount of Ca^2+^ available for release.^21^

### Blood flow and O_2_

Blood flow can bring oxygen necessary for aerobic ATP production and remove by-products of metabolic processes in working muscles, thus playing an important role in the maintenance of force output. Muscle voluntary contractions increase the mean arterial blood pressure,^22^ which consequently decreases the net blood flow to the working muscle and induces fatigue.^23^ The occlusion of blood flow to a working muscle substantially decreases the time to exhaustion ^24, 25, 26^ and increases the magnitude of the decline in force,^27, 28^ thus indicating the potential importance of blood flow in fatigue prevention. However, despite changes in blood flow accompanying the development of muscle fatigue, decreased blood flow does not seem to be a key factor in the development of fatigue. Wigmore *et al.*^29^ have used venous occlusion plethysmography to decrease blood flow of the ankle dorsiflexor muscles, and have found that the decline in MVC force precedes significant changes in blood flow to the muscle.

One of the important roles of blood flow is to provide O_2_ to the working muscles. It has been well documented that decreased oxygen availability to exercising muscle has profound consequences on muscle fatigue. Breathing hypoxic air can significantly increase muscle fatigue *in vivo*,^30, 31^ and enhanced O_2_ delivery to the exercising muscles^32^ directly attenuates muscle fatigue and increases muscle efficiency. However, O_2_ availability affects the fatigue process at moderate work intensities. Generally, oxygen uptake and ATP utilization are increased until the VO_2max_ is reached. During exercise at a very high intensity (usually the VO_2max_ is already reached), the demand for more ATP cannot be met by increases in oxygen delivery, thus resulting in an imbalance of metabolic homeostasis and leading to fatigue.^33^

### Energy

Muscular work must be supported by a ready supply of ATP energy. There are three major ATPases that require ATP for muscle activity: Na^+^/K^+^-ATPase, myosin ATPase and Ca^2+^ ATPase. The Na^+^/K^+^-ATPase pumps Na^+^ back out and K^+^ back into the fiber after an action potential. The myosin ATPase uses ATP to generate force and do work, and the Ca^2+^ ATPase pumps Ca^2+^ back into the SR, thus allowing for muscle relaxation. The activities of these enzymes account for 10%, 60% and 30% of total ATP use, respectively.^34^

Glycogen is the carbohydrate energy store for ATP production. There are three distinct subcellular localizations of glycogen: (1) intermyofibrillar glycogen, located between the myofibrils and close to SR and mitochondria; (2) intramyofibrillar glycogen, located within the myofibrils and most often in the I-band of the sarcomere; and (3) subsarcolemmal glycogen, located beneath the sarcolemma and primarily next to mitochondria, lipids and nuclei. Approximately 75% of the total glycogen store in the cells is intermyofibrillar glycogen.^35, 36^

It is a fundamental concept in exercise physiology that glycogen is an important fuel during exercise.^37^ As early as the 1960s, a strong correlation between muscle glycogen content and exercise endurance was found.^38^ When glycogen stores are limited, exercise cannot continue.^39^ Glycogen oxidation is a major source for ATP regeneration during prolonged exercise (>1 h) and high-intensity intermittent exercise.^40^ Furthermore, glycogen may be important because it produces tricarboxylic acid cycle intermediates, thus contributing to the maintenance of oxidative metabolism.^41^ Excitation-contraction coupling and relaxation have been reported to be affected by glycogen levels.^37, 42, 43^ Low-muscle glycogen and/or glycolytic-derived energy are associated with impaired SR Ca^2+^ release, reuptake, and Na^+^/K^+^-pump function.^43, 44^ However, how glycogen depletion affects the series of events and ultimately results in fatigue are not fully understood.

### Metabolic factors

Muscle contractions activate ATPases and promote glycolysis, thus leading to an increase in intracellular metabolites, such as H^+^, lactate, Pi and ROS, which contribute to the changes in cross-bridge activity.

Historically, H^+^ has been thought to have a role in the development of muscle fatigue. Glycolysis leads to the production of pyruvate, which feeds into the TCA cycle for oxidation. If pyruvate production exceeds its oxidation, excess pyruvate is converted into lactic acid, which dissociates into lactate and H^+^. The accumulation of H^+^ lowers the pH, thus potentially interfering with SR Ca^2+^ release, troponin C sensitivity to Ca^2+^ and cross-bridge cycling and resulting in impaired muscle force.^45^ However, the role of decreased pH as an important cause of fatigue is now being challenged.^46^ Several recent studies have shown that decreased pH may have little effect on contraction in mammalian muscle at physiological temperatures. Furthermore, there is a lack of association between changes in pH and MVC throughout fatiguing exercise and in recovery in humans.^47^

In addition to acidosis, anaerobic metabolism in skeletal muscle also involves hydrolysis of creatine phosphate (CrP) to creatine and Pi. The concentration of Pi can increase rapidly from approximately 5–30 mM during intense fatigue. Creatine has little effect on contractile function, whereas Pi, rather than acidosis, appears to be the most important cause of fatigue during high-intensity exercise.^48^ Increased Pi substantially impairs myofibrillar performance, decreases SR Ca^2+^ release and therefore contributes to the decreased activation.^49^

Mitochondrial respiration produces ATP and consumes O_2_, a process that generates ROS. The most important ROS include superoxide (O_2_•−), hydrogen peroxide (H_2_O_2_), and hydroxyl radicals (OH•). As the work intensity increases, ROS production increases. The most convincing evidence that ROS contribute to fatigue comes from experiments showing that pretreatment of intact muscle with a ROS scavenger significantly attenuates the development of fatigue. ROS affect muscle fatigue mainly through the oxidation of cell proteins such as the Na^+^–K^+^ pump, myofilaments, DHPR and RyR1,^50^ thus leading to the inhibition of SR Ca^2+^ release and myofibrillar Ca^2+^ sensitivity. In addition, ROS activate the group IV muscle afferents^51^ and directly inhibit motoneurons.

Other metabolites with probable roles in fatigue include ATP, ADP, PCr and Mg.^52^ For example, muscle ADP increases with intense contractile activity. In skinned fibers, ADP decreases fiber velocity but increases force, presumably because of more cross-bridges in the high force states. However, the more important role of ADP in eliciting fatigue appears to be related to the inhibition of the SR Ca^2+^ pump and the resulting disturbances in ECC rather than direct effects on the cross-bridge.^53^

### Fatigue reactants

Organisms have different levels of adaptive responses to fatigue stress, including the CNS nervous system, sympathetic nervous system, endocrine system (hypothalamus-pituitary-adrenal axis, HPA axis), and innate immune system (that is, non-specific cytokines, complement system and natural killer cells). Many fatigue reactants, such as cortisol, catecholamine, IL-6 and HSPs, may have roles in muscle function.^54^

HSPs are involved in the adaptation to fatigue stress. Within the family of HSPs, HSP25 protein is abundantly expressed in skeletal muscle and increases with muscle contractile activity.^55^ Interestingly, Jammes *et al.* have reported that a widespread HSP25 response to fatigue in a single hindlimb muscle is responsible for a global adaptive response to acute localized stress and have demonstrated that group III and IV muscle afferents play an important role in the fatigue-induced p-HSP25 response; moreover, the sympathetic nerve supply to the muscles and kidney comprises the efferent arm of the p-HSP25 activation.^56^ Skeletal muscle HSP25 has been reported to stabilize muscle structure and repair damaged muscle proteins,^57^ as well as to decreases apoptosis in cultured muscle C2C12 cells by inhibiting the intrinsic and extrinsic apoptotic cell death pathway.^58^

Orosomucoid (ORM) is an acute-phase protein, with a very low pI of 2.8–3.8 and a very high carbohydrate content of 45%. It is predominantly synthesized in the liver, and many extra-hepatic tissues have also been reported to produce ORM under physiological and pathological stress.^59^ Our studies have found that the expression of ORM is markedly increased in the serum, liver and skeletal muscle in response to various forms of fatigue, including sleep deprivation, forced swimming and treadmill running. Interestingly, exogenous ORM increases muscle glycogen and enhances muscle endurance, whereas ORM deficiency results in decreased muscle endurance, thus indicating that ORM is an endogenous anti-fatigue protein. Further studies have demonstrated that ORM binds to C–C chemokine receptor type 5 (CCR5) on muscle cells and activates AMPK, thus promoting glycogen storage and enhancing muscle endurance, and representing a positive feedback mechanism for resisting fatigue and maintaining homeostasis.^60, 61^ Modulation of the level of ORM and CCR5 signaling may be a novel strategy for the management of muscle fatigue.

## Non-invasive techniques for the ASSESSMENT OF sites of muscle fatigue

Muscle fatigue is manifested most naturally in the intact organism. Non-invasive techniques of site-specific stimulation can now be used to evaluate the potential sites of the entire system for force production in human studies. All evoked muscle responses are recorded via electromyography (EMG) electrodes placed on the muscle.

### Transcranial magnetic stimulation

Transcranial magnetic stimulation involves applying magnetic stimulation to the motor cortex and is optimized to activate the muscle of interest.^1^ The stimulation-induced muscular response recorded by EMG is known as the motor-evoked potential (MEP). MEP is influenced not only by cortical excitability but also by spinal cord motor neuron excitability and muscle factors. MEP depression can occur in the relaxed muscle after a fatiguing exercise, possibly as a result of afferent input from the fatigued muscle. MEP is increased in the upper- and lower-limb muscles during sustained submaximal isometric contractions and is regarded as an augmentation of the central drive to the lower motoneuron pool that allows a constant level of force to be maintained despite the development of peripheral fatigue. During sustained MVC, MEP has been reported to increase during the first seconds and then to level off, increase linearly or remain stable, depending on the protocol used (that is, continuous vs intermittent) and the muscle investigated.^1^

### Cervicomedullary region electrical stimulation

Electrical stimulation in the cervicomedullary region aims to activate the corticospinal tract at a subcortical level, thereby eliminating cortical contributions to the evoked muscle response. The muscular response recorded by EMG is known as the cervicomedullary motor-evoked potential (CMEP). Comparison of MEP and CMEP is helpful for the localization of excitability at the cortical or subcortical level. During a sustained 30% MVC of the plantar flexors, a large increase in MEP and only a slight increase in CMEP have been reported, thus suggesting a small contribution of spinal factors to the increase in corticospinal excitability during submaximal fatiguing contractions. In contrast, during 50% MVC of the elbow flexors to task failure, similar MEP and CMEP kinetics has been found, thus indicating that central changes occur almost entirely at the spinal level.^62, 63, 64^

### Peripheral nerve low-intensity electrical stimulation

Low-intensity electrical stimulation of the peripheral nerve preferentially activates the Ia sensory fibers, which synapse with the α-motoneuron in the spinal cord. The signal is then carried along the motor neurons to the muscle, generating a response in the muscle known as the Hoffmann reflex (H-reflex). The H-reflex is used to assess spinal excitability and inhibition. Although there are several of an increase^65^ or no change,^66^ the general consensus is that there is an overall decline in the amplitude of the H-reflex with the development of muscle fatigue, thus indicating a decrease in spinal excitability.^67, 68^ The rate and degree of decrease in H-reflex amplitude appear to be dependent on the type of fatiguing task.

### Peripheral nerve high-intensity electrical stimulation

High-intensity stimulation of the peripheral nerve directly activates the α-motoneuron, evoking a motor response (m-wave) from the muscle. The m-wave is a compound action potential recorded with surface EMG and is used to assess peripheral excitability of the muscle membrane and transmission at the neuromuscular junction. A change in the twitch force without a change in the m-wave indicates a failure of excitation-contraction coupling.

Short-duration fatiguing contractions (~20 s) induce an enhancement in the amplitude and area of the m-wave.^69^ A longer (4-min) sustained maximal contraction does not induce changes in the amplitude of the m-wave^70^ but results in a significant decline in the central activation, thus suggesting that central factors contributing to fatigue can occur in the absence of a peripheral change in membrane excitability. However, more longer-duration contractions that induce fatigue (~17 min) can also induce a decline in the muscle membrane excitability and m-wave size.^69^

## Biomarker for the diagnosis of muscle fatigue

At present, there are still no specific factors that have been consistently associated with a particular type of fatigue. Exercise types (for example, aerobic/anaerobic, short or long term), contraction type (for example, incremental/constant, isometric/non-isometric, concentric/eccentric), and fatigue degree and duration all affect the biomarker profile. According to the mechanism and metabolic changes during muscle fatigue, three categories of biomarkers have been determined: (1) ATP metabolism biomarkers, such as lactate, ammonia and hypoxanthine; (2) Oxidative stress biomarkers (ROS), such as lipid peroxidation, protein peroxidation, and antioxidative capacity; and (3) Inflammatory biomarkers, such as TNF-α, leukocytes, and interleukins.^71^

### ATP metabolism biomarkers

Under normal circumstances, the total adenine nucleotide pool (ATP+ADP+AMP) remains constant. When the ATP supply fails to meet the consumption of ATP during exercise, fatigue occurs. To maintain the ATP/ADP ratio, two molecules of ADP may be converted to one molecule of ATP and one molecule of AMP. AMP is subsequently degraded by AMP-deaminase to IMP and ammonia.^72^ IMP is degraded to inosine and hypoxanthine, and ammonia is further converted to urea nitrogen (BUN), thus increasing blood BUN. In the case of inadequate oxygen supply, oxidative phosphorylation of ADP to generate ATP fails to meet the energy requirement, and the ATP production shifts from aerobic processes (the processing of glucose/glycogen, lipids or amino acids) to anaerobic glycolysis or glycogenolysis,^73^ thereby resulting in lactate accumulation. The best-known biomarkers of muscle fatigue from ATP metabolism include lactate, ammonia, and hypoxanthine.^74, 75^ Lactate and ammonia are usually determined in the serum. Hypoxanthine is usually analyzed in the serum or urine.

Serum lactate increases with exercise intensity in healthy and diseased subjects.^76^ However, serum lactate does not appear to be related to age, sex, and physical fitness. Under the conditions of workload standardization, serum lactate appears to be a promising biomarker of muscle fatigue.^73^ Serum ammonia closely follows the lactate response during exercise ^73^ and increases during exercise. Serum ammonia is not associated with age^77^ and remains low in physical fitness, but is higher in men than in women.^78^ Serum hypoxanthine significantly increases immediately after exercise.^79^ There exists a sex difference ^80^ but a lack of reliable data on age- or physical fitness-dependency on serum hypoxanthine.

### Oxidative stress biomarkers

Reactive oxygen species (ROS) remain at a low level in resting skeletal muscle but increase in response to contractile activity. ROS products lead to protein, lipid or nucleic acid oxidation accompanied by a marked decrease in the antioxidant capacity,^81^ thus ultimately inducing fatigue. Promising biomarkers to assess oxidative damage in muscle fatigue include lipid peroxidation biomarkers (that is, thiobarbituric acid-reactive substances (TBARS) and isoprostanes), and protein oxidation biomarkers (that is, protein carbonyls (PCs). Biomarkers to evaluate the antioxidant capacity include glutathione (GSH), glutathione peroxidase (GPX), catalase, and the total antioxidant capacity (TAC).^71^

TBARS are indicators of lipid peroxidation and oxidative stress, which form during the decomposition of lipid peroxidation products that react with thiobarbituric acid and form a fluorescent red adduct. Isoprostanes are prostaglandin-like compounds derived from the peroxidation of essential fatty acids catalyzed by ROS. PCs are mainly derived from the oxidation of albumin or other serum proteins and are regarded as markers of oxidative protein injury. GSH is a pseudotripeptide that is present in nearly all cells and plays an important role in ROS scavenging. GPX and catalase are both enzymes that scavenge hydrogen peroxide into water and oxygen. TAC is defined as the sum of the antioxidant activities of the nonspecific pool of antioxidants.

TBARS, PC, catalase and TAC are usually determined in the serum, but TBARS are also detectable in the saliva. Isoprostanes are usually measured in the serum, urine, or other body fluids and blood cells. GSH and GPX are present in cells and are detectable in serum and saliva.^82^ With increasing exercise intensity, the levels of TBARS, isoprostanes, PC, catalase, TAC and GPX all increase, and that of GSH decreases.^76, 82, 83, 84^ With age, the levels of TBARS, isoprostanes and TAC increase,^85, 86, 87^ those of GSH, GPX and catalase decrease,^88, 89, 90^ and changes in PC remain controversial.^91, 92^ With physical fitness, the levels of TBARS, PC, GSH and GPX increase,^93^ whereas the changes in catalase, PC and TAC still lack definite data.^94^ The levels of TBARS, isoprostanes, PC, catalase and TAC have been reported to be lower in females than in males,^90, 95, 96, 97^ whereas GSH and GPX levels show an opposite trend.^89, 98^

### Inflammatory biomarkers

In addition to the depletion of ATP and ROS production, exercise and fatigue also induce local or systemic inflammatory reaction. Promising biomarkers to evaluate inflammation in muscle fatigue include leukocytes, IL-6 and TNF-α.^71^

T-lymphocytes, especially CD4+ and CD8+ lymphocytes, are mobilized from peripheral lymphoid compartments into the blood after exercise.^99^ In addition, neutrophils show a significant increase immediately after exercise. These changes represent a nonspecific immune response induced by ischemia in a stressed tissue, while there is a lack of a real injury.^100^ IL-6, acting as an important pro-inflammatory (monocytes and macrophages) cytokine, is also now regarded as one of myokines released from muscle in response to contractions.^101^ The levels of TNF-α, predominantly produced by macrophages, also increase as a result of muscle fatigue. Generally, IL-6 and TNF-α levels are determined in the serum. IL-6 levels can also be determined in the saliva.

With age, the change in T-cells expressing CD8 remains controversial,^102, 103^ whereas the change in IL-6 is age independent. Sex differences in T-cell immune responses are particularly evident in graft-versus-host disease, with a stronger effect in females,^104^ and IL-6 levels are also markedly lower in females.^102^ TNF-α levels appear to be independent of age, sex and physical condition.

There are still many potential immunological biomarkers, including C-reactive protein (CRP), IL-8, IL-10, IL-15, HSP27, HSP70, plasma DNA and orosomucoid (ORM).^72, 101, 105^ For example, IL-15 has been found to accumulate within the muscle after regular training.^106^ ORM, an acute-phase protein with immune-modulating activity, significantly increases in serum, muscle and liver tissues in response to various forms of muscle fatigue in rodents.^60^ Of course, there are still several biomarkers that are unsuitable for the diagnosis of muscle fatigue, such as elastase, IL-1β and complement C4a, because their concentrations do not change substantially after exercise.^107^

## Potential treatment for muscle fatigue

Improper exercise, long time combat, military training and some related diseases (for example, cancer and stroke) can cause muscle fatigue, which negatively affects athletic achievement, military combat ability and patient recovery. At present, there are still no official or semi-official recommendations for the treatment of muscle fatigue. However, some nonspecific treatments, such as synthetic products (for example, amphetamine and caffeine), natural products (for example, American ginseng and rhodiola rosea) and nutritional supplements (for example, vitamins and minerals and creatine), have been used clinically or experimentally, and have shown some effects in various studies.

### Synthetic products

Amphetamine, ephedrine, caffeine, for example, are all synthetic products that excite the central nervous system or sympathetic nervous system and promote resistance to muscle fatigue. Almost half of the stimulant abuse in sport involves amphetamines and ephedrine, as reported by WADA (World Anti-Doping Agency) in 2005. The use of amphetamines, amphetamine derivatives, propanolamine and ephedrine remains illegal in competition. However, caffeine and pseudoephedrine have been accepted at any level since 2004.

#### Amphetamine

Amphetamine is a phenethylamine-type stimulant and antidepressant that is highly addictive and produces euphoria and an elevated mood. Amphetamine at low to moderate doses enhances the physical performance of humans and animals.^108, 109, 110^ However, the underlying mechanism remains largely unknown. High body temperature is one of the strongest exhaustion signals. Recently, Morozova E has reported that amphetamine may mask or delay fatigue in rats by slowing down the exercise-induced elevation in core body temperature. Although amphetamine usage is prohibited during competitions, it may be used in some situations, such as in combat, to improve performance by delaying exhaustion.^111^

#### Caffeine

The use of caffeine as a sports-related enhancement drug is well documented. High caffeine dose consumption enhances performance during extended periods of exercise.^112, 113^ Indeed, the performance-enhancing effects of caffeine have been described for both prolonged aerobic exercises and prolonged activities involving resistance.^114^ The effects of caffeine on short periods of intense aerobic activity (5–30 min) have been reported to be significantly beneficial, but its effects on very short-term anaerobic exercise, for example, sprinting, are inconclusive.^115^ Mechanistically, caffeine has been reported to increase the epinephrine and norepinephrine response associated with exercise.^116^ In addition, caffeine potentiates muscle contractility via the induction of SR calcium release, inhibition of phosphodiesterase isoenzymes, inhibition of glycogen phosphorylase enzymes and stimulation of the sodium/potassium pump.^115^

#### Others

Other sympathomimetic stimulants, such as ephedrine, pseudoephedrine and phenylpropanolamine, are several times less potent than amphetamines in improving performance.^116, 117, 118^ Bell *et al.*^119^ have provided clear evidence that ephedrine at a high dose improves endurance exercise in subjects running 10 km. In addition, taltirelin, a synthetic thyrotropin-releasing hormone (TRH) analog, effectively improves sports activity.^120^ Cocaine, which causes a rapid sympathetic response, significantly increases endurance during high-intensity exercise.^121^ Modafinil, a new drug type that acts on the central nervous system and keeps subjects awake,^122^ markedly prolongs exercise time to exhaustion ^123^ and has been widely used in the war to allow people to resist fatigue. Benzamide derivatives, such as 1-(1, 3-benzodioxol-5-ylcarbonyl) piperidine (1-BCP), significantly prolong the time of forced swimming in mice, through an unclear mechanism.^124^

### Natural products

More than half of the drugs introduced worldwide are derived from or are inspired by natural products. In the past few decades, health scholars and athletic physiologists have been searching for natural products that can improve athletic ability and resist or eliminate fatigue in human beings. Now, more and more natural products and their extracts have been revealed as potentially anti-fatigue agents.

#### Araliaceae ginseng species

American ginseng, panax ginseng C. A. Meyer and radix notoginseng all belong to the araliaceae ginseng species. American ginseng is the root of panax quinquefolium, which is currently grown in Canada and eastern USA. Panax ginseng C.A. Meyer. (ginseng) is an edible and medicinal Chinese herb that is often used in Asian countries. Panax notoginseng (Burk.) F.H. Chen is cultivated throughout Southwest China, Burma, and Nepal. The root, a commonly used part of this plant, is called radix notoginseng or Sanchi. All of them contain multiple active components, such as saponins, polysaccharides, flavonoids, vitamins and microelements, which are responsible for the effects in the improvement of physical fatigue in humans and animals. For example, saponins or protein extracted from American ginseng significantly lengthens the swimming time in mice via increasing the levels of liver glycogen and muscle glycogen.^125^ Polysaccharides, Ginsenoside Rb1, Ginsenoside Rg3 or small molecule oligopeptides, derived from Panax ginseng C. A. Meyer, have all been reported to have marked anti-fatigue activity in mice swimming or grasping test.^126, 127, 128^ One particular type of ginseng, red ginseng, has been found to have a positive effect on sports performance in 11 volunteers undertaking repetitive anaerobic exercise.^129^ Multiple mechanisms are involved in the anti-fatigue effects of panax ginseng C. A. Meyer, including enhancing lactate dehydrogenase (LDH) activity, increasing hepatic glycogen levels, retarding the accumulation of serum urea nitrogen (SUN) and blood lactic acid (BLA), inhibiting oxidative stress and improving mitochondrial function in skeletal muscles. Regarding panax notoginseng, a single dose has been reported to enhance aerobic capacity, endurance and mean blood pressure (MAP) in young adults.^130^ Total saponins extracted from panax notoginseng, the principal active ingredients, have been found to extend the exhaustive swimming time of mice, delay the increase in lactate in the blood, and increase the tissue glycogen content.^131^

#### Rhodiola rosea

Rhodiola rosea (R. rosea), belonging to the family Crassulaceae and genus Rhodiola, is a commonly used plant in folk medicine in Eastern Europe and China. It is also an important resource against fatigue. The ingredients of rhodiola rosea include salidroside and rosavin. Rosavin is the only constituent unique to R. rosea from the Rhodiola genus, and salidroside is common to most other Rhodiola species. The natural ratio of rosavins to salidrosides in R. rosea is approximately 3:1. Salidroside has been identified as the main anti-fatigue ingredient in Rhodiola rosea. Acute intake of Rhodiola rosea containing 3% rosavin+1% salidroside plus 500 mg starch has been found to improve endurance exercise capacity in young healthy volunteers.^132^ Fermented R. rosea extract has also been found to significantly increase swimming time, hepatic superoxide dismutase content, and serum lactate dehydrogenase in mice.^133^

#### Garlic

Garlic (*Allium sativum*) is an herb that is used mainly as a food in many countries. Garlic was given to soldiers and athletes as a tonic in ancient Rome. Recently, the anti-fatigue effect of garlic has been reported by many researchers. Garlic-processing methods affect the anti-fatigue effects.^134^ The main methods for processing raw garlic can be classified as (1) production of garlic powder, obtained after the drying of raw garlic; (2) production of garlic oil, distilled by steaming raw garlic; (3) production of oil macerate, extracted from raw garlic with vegetable oil; and 4) production of aged garlic extract (AGE).^135^ Ushijima *et al.* have examined the effect of raw garlic juice, heated garlic juice, dehydrated garlic powder and AGE on physical strength and recovery from fatigue. They have found that raw garlic and AGE prolongs the treadmill running time of mice and enhances the speed of recovery of rectal temperature after immersion in cool water. These effects are related to the improvement of peripheral circulation, an action of anti-stress, and improvement of nutrition.^136^ Recently, clinical studies have revealed many intriguing findings.^137^ Verma *et al.* have investigated the effects of garlic oil on cardiac performance and exercise tolerance in 30 patients with coronary artery disease. After an initial treadmill stress test, the subjects were administered garlic oil for 6 weeks, and treadmill stress tests were repeated. In comparison with the initial test, garlic significantly decreased the heart rate at peak exercise and work load on the heart, thus leading to the better exercise tolerance.

#### Others

Enhancing the energy metabolism effectively helps to improve exercise capacity. Chinese yam and fructus aurantii have been reported to improve muscle glycogen, liver glycogen and other indicators.^138, 139^ Increasing numbers of natural products and their active components have been reported to have certain curative effects against physical fatigue, such as ophiopogon root, astragalus, Chinese wolfberry, caltrop, *Acanthopanax giraldii*, *Cordyceps sinensis*, *Ganoderma lucidum*, eucommia, *Ginkgo biloba*, radix paeoniae alba, gynostemma, acanthopanax, angelica, radix rehmanniae and radix polygoni multiflori. However, most of them still require extensive studies to determine their anti-fatigue effects and mechanisms.

### Nutritional supplements

Several nutritional factors that may limit exercise performance have been identified, thus leading to the widespread use of nutritional strategies. Nutritional supplementation is regarded as legal by the International Olympic Committee (IOC) and, therefore, has gained popularity as a way to achieve performance enhancement. Nutritional supplements can be grouped into dietary supplements (for example, multivitamins, fish oils and glucosamine sulfate/chondroitin), ergogenic aids (for example for example, protein powder/amino acids and creatine) and sports foods (for example, sports drinks and meal replacement).^140^ The most commonly used products are sports drinks and vitamin/mineral supplements, followed by creatine and protein supplements.^141^

#### Vitamins and minerals

Despite their relative paucity in the diet and the body, vitamins and minerals are key regulators of health and function, including work performance. They are not direct sources of energy but facilitate energy metabolism. Water-soluble vitamins include B vitamins (thiamin, riboflavin, niacin, pyridoxine, folate, biotin, pantothenic acid, vitamin B12 and choline) and vitamin C. Fat-soluble vitamins include vitamin A, D, E, and K. Vitamin A, C and E are also antioxidants. Twelve minerals are designated essential nutrients. Magnesium, iron, zinc, copper and chromium have the potential to affect physical performance.^142^ Researchers have shown that vitamin and mineral deficiencies may result in decreased physical performance, and their supplementation improves physical performance in persons with preexisting deficiencies. For example, severe deprivation of folate and vitamin B12 result in anemia and decrease endurance work performance. Iron supplementation improves progressive fatigue resistance in iron-depleted, nonanemic women.^143^ However, the use of vitamin and mineral supplements does not appear to improve performance in people consuming adequate diets.^142^ Dietary supplementation in athletes at the Australian Institute of Sport for up to 8 months, including vitamins B1, B2 (riboflavin), B6, B12, C, E, A, folate and copper, magnesium, zinc, calcium, phosphorus, as well as aluminum, has not been found to improve athletic performance.^144^

#### Fish oil

Fish oil, a dietary supplement, has been shown to have beneficial effects on performance. Fish oil is rich in omega-3 fatty acids, specifically docosahexaenoic acid (DHA) and eicosapentaenoic acid (EPA), which have been found to improve cardiac energy efficiency, fat metabolism and immunomodulatory responses. The consumption of fish oil (containing 1050 mg EPA+750 mg DHA) for 3 weeks in 20 healthy subjects has been found to decrease the body fat percentage and improve exercise performance and physiological recovery after exercise.^145^

#### Creatine

Creatine (Cr), a nitrogen-containing compound synthesized in the body from glycine, arginine and methionine, is also found in the diet, primarily in red meat and seafood. The creatine/phosphorylcreatine system can provide energy when the rate of ATP utilization is higher than the rate of production by mitochondrial respiration, thus maintaining ATP homeostasis.^146^ Introduced to the general public in the early 1990s, creatine has become one of the most widely used nutritional supplements or ergogenic aids, and has been consistently shown to increase performance in high-intensity intermittent exercise.^147^ Creatine is regarded as legal by the International Olympic Committee. Therefore, creatine supplementation is a potential ergogenic strategy to improve muscle endurance.

#### Red bull

Red bull contains a mixture of carbohydrates, taurine, glucuronolactone, vitamin B and caffeine, and it is a commonly used energy drink. Several small studies have reported that carbohydrate and caffeine consumption improves aerobic and anaerobic performance as well as cognitive functions such as concentration, alertness and reaction time.^148^ It has been postulated that the effects are from the modulation of adenosinergic receptors by caffeine and taurine.

#### Others

Carnitine plays an essential role in fatty acid oxidation in muscle. However, there is a lack of definite evidence regarding its beneficial role in performance as a supplement. Protein supplements have been demonstrated to be ineffective except in rare cases in which dietary protein intake is inadequate. Individual amino acids, especially ornithine, arginine and glutamine, are also commonly used as supplements. However, their effects on performance are not supported by documented evidence. Acute-phase protein ORM has been reported to enhance muscle endurance after vein or intraperitoneal injection in rodents,^60^ but it is not convenient for daily supplementation. In theory, the use of antioxidant vitamins and glutamine during periods of intensive training should be beneficial, but further evidence is still needed before they are recommended as supplements.^149^

## Conclusions

Muscle force production involves a sequence of events, extending from cortical excitation to motor unit activation to excitation–contraction coupling, and ultimately leading to muscle activation. Changes at any level in this pathway, including changes in the nervous, ion, vascular, and energy systems, impair force generation and contribute to the development of muscle fatigue. Metabolic factors and fatigue reactants, such as H^+^, lactate, Pi, ADP, ROS, HSP25 and ORM, also affect muscle fatigue. Site-specific stimulation via non-invasive techniques provides a method to gain systemic insight into the fatigue process under physiological conditions. Although there is a lack of consensus, a sex- and age-specific distribution in muscle fatigue has been observed, in which children, older adults and males are more resistant to fatigue than adults and females. Biomarkers of ATP metabolism, oxidative stress and inflammatory reactions are helpful for the diagnosis of muscle fatigue. Despite the lack of official or semi-official recommendations, muscle fatigue has been reported to be improved by some nonspecific treatments, including CNS-exciting drugs, natural products and nutritional supplements. More potential mechanisms, biomarkers, targets and related drugs for muscle fatigue— for example, ORM—still need to be explored in the future.

## Publisher’s note

Springer Nature remains neutral with regard to jurisdictional claims in published maps and institutional affiliations.
